# Comparison of Clinical Characteristics, Therapy, and Short-Term Prognosis between Blunt and Penetrating Abdominal Trauma: A Multicentric Retrospective Cohort Study

**DOI:** 10.1155/2024/5215977

**Published:** 2024-02-13

**Authors:** Yi Liu, Yunhe Gao, Zhida Chen, Jianxin Cui, Wenquan Liang, Ze Wang, Linde Sun, Chuan Pang, Yuan Lv, Guoxiao Liu, Tingting Lu, Gan Zhang, Xiaoyu Dong, Hong Xu, Sheng Yao, Feng Liang, Gang Liu, Gang Chen, Jianmiao He, Wentong Xu, Bo Wei, Hongqing Xi, Lin Chen

**Affiliations:** ^1^Department of Abdominal Trauma Surgery, The First Medical Center of Chinese PLA General Hospital, Beijing 100853, China; ^2^Department of Gastric Surgery, The First Medical Center of Chinese PLA General Hospital, Beijing 100853, China; ^3^Research Institute of General Surgery, The First Medical Center of Chinese PLA General Hospital, Beijing 100853, China; ^4^Department of General Surgery, The Fifth Medical Center of Chinese PLA General Hospital, Beijing 100039, China; ^5^Department of General Surgery, The Seventh Medical Center of Chinese PLA General Hospital, Beijing 100007, China; ^6^Department of General Surgery, The Third Medical Center of Chinese PLA General Hospital, Beijing 100039, China; ^7^Department of General Surgery, The Fourth Medical Center of Chinese PLA General Hospital, Beijing 100048, China; ^8^Department of General Surgery, The Sixth Medical Center of Chinese PLA General Hospital, Beijing 100048, China; ^9^Department of General Surgery, The Eighth Medical Center of Chinese PLA General Hospital, Beijing 100091, China

## Abstract

**Objective:**

Large-scale studies on the characteristics and management of abdominal trauma in megacities in China are lacking. The aim of this study was to analyze and present the clinical patterns and treatment status of abdominal trauma in regional medical centers.

**Methods:**

Cases of abdominal trauma treated at seven medical centers in Beijing from 2010 to 2021 were collected. Clinical information about age, sex, injury cause, geographic distribution, abbreviated injury scale/injury severity score (AIS/ISS) value, injury-hospital time, preoperative time, surgically identified organ injuries, type of surgery, causes of reoperation and 90-day mortality was included in this study. Clinical characteristics, treatment methods, and short-term prognoses (90-days survival) were compared between blunt abdominal trauma (BAT) and penetrating abdominal trauma (PAT) cases. Non-normally distributed data are described as medians (IQR), and the Mann‒Whitney *U* test was performed; qualitative data were analyzed using the *X*^2^ test. Univariate and multivariate survival analyses were performed by the Cox proportional hazards model.

**Results:**

A total of 553 patients (86.98% male) with a median age of 36.50 (27.00–48.00) years were included. The BAT group had a significantly higher proportion of serious injury (*P*=0.001), lower initial hemoglobin level (*P*=0.001), and a lower laparoscopy surgery rate (*P*=0.044) compared to the PAT group. Additionally, more BAT cases were from the area around Beijing (*P*=0.008) and a longer injury-regional hospital time (10.47 (5.18–22.51) hours vs. 7.00 (3.80–15.38) hours, *P*=0.001). In the hollow viscus injury subgroup, the BAT group had a significantly longer injury-regional hospital time and preoperative time compared to the PAT group (injury-regional hospital time: 10.23 (6.00–21.59) hours vs. 7.07 (3.99–13.85) hours, *P*=0.002; preoperative time: 3.02 (2.01–5.58) hours vs. 2.81 (1.85–3.63) hours, *P*=0.047). The overall 90-day mortality was 11.9%, and longer injury-regional hospital time (HR: 1.01, 95% CI: 1.00–1.02, *P*=0.008), receipt of ICU treatment (HR: 4.69, 95% CI: 2.54–8.65, *P*=0.001), and severe ISSs (ISS > 25 vs. ISS < 16, HR: 2.78, 95% CI: 1.38–5.601, *P*=0.004) had a worse impact on survival.

**Conclusion:**

More patients with BAT were transferred to higher-level hospital, leading to significantly longer prehospital and preoperation time. In the subgroup of hemodynamically stable individuals, more patients with BAT experienced hollow viscus injuries. For those patients, aggressive diagnostic laparoscopic exploration may be beneficial. Patients with longer injury-regional hospital intervals, the need for ICU care, and higher injury severity scores (ISSs) suffered from worse prognoses.

## 1. Background

Trauma is the leading cause of death among young and middle-aged populations in modern society [1]. The abdomen is the third most common trauma site, accounting for approximately 5%–6% of all traumatic injuries in peacetime and approximately 8%–10% in wartime [2–4], only next to head and limb trauma. Although the overall mortality rate for war wounds has decreased to 10% in recent conflicts, abdominal trauma, especially penetrating abdominal trauma, still has high morbidity and mortality [5]. The blunt abdominal trauma (BAT) is the most common type of abdominal trauma. In individuals with BAT, liver and spleen injuries are the most common injuries, and the reported rate of occurrence of hollow and mesenteric injuries ranges from 3%–6% [6]. Unlike BAT, the major cause of the penetrating abdominal trauma (PAT) is stab injury, and small-intestinal and colonic injuries are the most common injuries to organs [7]. Exploration laparotomy is a recognized treatment modality for PAT [8, 9]. However, for BAT, diagnosis and treatment can be difficult, especially for asymptotic hollow organ injuries. Most solid organ injuries, including 80% of liver and spleen injuries, are amenable to interventional radiation treatment or symptomatic treatment [10]. However, for asymptotic hollow organ injuries, diagnosis by physical examination or imaging examination is sometimes difficult, and the reported missed or misdiagnosis rate is 30%–40% [3, 11]. Delayed diagnosis or operation is also reported to be associated with an increased rate of sepsis, longer hospital stays, and increased mortality risk. According to our experience, the proportion of hollow viscus injuries is higher than that in previous reports in China, and the clinical characteristics of civil abdominal trauma may be quite different from those in Western countries due to the large variations in injury causes and medical systems. Multicenter, large-sample abdominal trauma data from megacities are needed to describe and analyze the current status of the treatment and features of abdominal trauma.

## 2. Methods

### 2.1. Selection Criteria

This study was approved by the Chinese PLA General Hospital Ethics Committee, reference number S2022-124-01. In this study, 1699 abdominal trauma patients who had been treated in the First to Eighth Medical Center of Chinese PLA General Hospital from January 1, 2010, to December 30, 2021, were initially screened. By applying the inclusion and exclusion criteria, a total of 553 patients were selected. The inclusion criteria were as follows: (1) age ≥14 years, with a primary diagnosis of abdominal trauma, with or without injuries to other anatomic parts; (2) admission for another diagnosis but eventual diagnosis with abdominal trauma; (3) a diagnosis confirmed by imaging or surgery. The exclusion criteria were as follows: (1) Cases with insufficient clinical information that would affect the statistical analysis and (2) patients who were discharged after a period of observation only, without requiring any specialized medical interventions. The flowchart of the selection procedure is shown in Figure 1.

### 2.2. Clinical Definitions

All data sources utilized in this project were derived from a multicenter database specifically focused on abdominal trauma. To ensure the reliability of clinical information, essential entries and information were carefully defined and subsequently collected, including general patient data and injury course; perioperative examination; first and final diagnosis; and surgical, recovery and prognosis data.

The prehospital transit time was defined as the time from injury to primary hospital admission. The injury-regional hospital time was defined as the time from injury to admission to one of the regional medical centers included in this study. The preoperative time referred to the interval between the time of admission to the regional hospital and the beginning of surgery. Injury types or causes were classified as traffic accident injury, high-fall injury, mechanical injury, sharp-object injury, fall injury, firearm injury, and other violent injuries. The abbreviated injury scale/injury severity score (AIS/ISS) was used to score the injury severity [12, 13]. The abdominal AIS score was required in all patients, and the ISS was required only in patients with multiple anatomic injuries. Injury severity was independently scored by two trauma surgeons (Yi Liu and Zhi-da Chen); when opinions were inconsistent, disagreement was resolved by referral to another senior consultant (Hong-qing XI). The initial systolic blood pressure of 90 or higher, without the need for fluid resuscitation, is indicative of hemodynamic stability.

In this study, we categorized surgical interventions into the following types: (1) repair, including gastrointestinal tract repair, mesenteric, and omental repair, hepatorrhaphy, splenorrhaphy, etc.; (2) resection, including gastrointestinal resection and anastomosis, hepatectomy, splenectomy, etc.; (3) neostomy, including small intestinal stoma formation and transverse colon and sigmoid colostomy; and (4) other surgical methods, including interventional therapy, debridement, catheter drainage, etc. Regarding the statistics on injured organs, only the injured organs confirmed by operation were counted, while the imaging-diagnosed organs are not included in Table 1.

### 2.3. Statistical Methods

Statistical analysis and plotting were performed using SPSS Statistics 26.0 and GraphPad Prism 9 software. Data were tested for normal distribution by the Kolmogorov‒Smirnov test. Normally distributed variables (measurement data) are described as the mean ± variance, and a *t* test or analysis of variance was performed for difference analysis. Non-normally distributed data are described as the median (interquartile range, IQR), and the Mann‒Whitney *U* test was performed for difference analysis. Enumeration data are expressed as cases (%), and the *X*^2^ test or Fisher's exact test was performed for difference analysis. The short-term (90 days) survival analysis was conducted by the Cox proportional hazards model. We used univariate analysis to explore the potential prognostic factors and put factors with *P* < 0.10 into multivariate Cox regression. All tests were two sided, and significant differences were considered when *P* < 0.05.

## 3. Results

### 3.1. Patient Baseline Data

A total of 553 patients were included in this study, with a preponderance of males (481, 86.98%) at a median age of 36.5 years (IQR: 27.00–48.00 years). As shown in Table 2, the patients with abdominal trauma were mainly young and middle-aged, and the 18- to 44-year-old population was the largest group, accounting for 61.31% of the total patients. Blunt abdominal trauma (BAT) was more commonly seen, with a total of 383 patients (69.26%). Compared with those with BAT, patients with penetrating abdominal trauma (PAT) were significantly younger (BAT: 39 years (28.00–50.00 years) vs. PAT: 33 years (33.00–44.00 years), *P*=0.001). Comparison of vital signs and laboratory results showed no significant differences in initial systolic blood pressure (SP), heart rate, lactate level, and potential of hydrogen value (PH) between the two groups. However, the initial hemoglobin level (HE) was significantly lower in the BAT compared to the PAT (BAT: 118 g/L (99.00–139.00 g/L) vs. PAT: 130 g/L (111.50–147.00 g/L), *P*=0.001).

Compared with the first six calendar years, the number of patients from areas surrounding Beijing significantly decreased in 2016–2021 (*P*=0.001), as shown in Figure 2. Significantly more patients with BAT than those with PAT were transported from areas surrounding Beijing (*P*=0.008).

### 3.2. Injury Causes and Damaged Organs

As shown in Table 2, traffic accident injury was the main injury cause, accounting for 40.69% (225 patients), and it was also the most common injury cause in BAT patients, accounting for 57.44%. The second most common injury cause was sharp-object injury, accounting for 24.77% (137 patients), which was the most common injury cause in PAT patients. The third most common injury cause was high-fall injury (71 patients, 12.84%). In the comparison of injured organ subgroups among patients with hemodynamically stable conditions, patients with hollow viscus injuries showed a significantly higher proportion in the BAT group compared to the PAT group (*P*=0.001). In terms of the injured organs listed in Table 1, the liver (22.30%) and spleen (22.67%) were the most frequently injured targets in abdominal trauma patients, and hollow viscus injury accounted for 33.46% of all organ injuries. In BAT patients, the spleen (28.18%), liver (25.44%), and small intestine (14.71%) were the three most frequently impaired organs. In PAT patients, the most frequently injured organs were the small intestine (23.29%), colon and rectum (19.86%), and stomach (16.44%).

### 3.3. Trauma Severity Score

In this study, multiple injuries accounted for the majority, with a total of 375 patients (67.81%). The severity of abdominal trauma was evaluated with the AIS score. Among the patients, a total of 61 patients had severe abdominal injury (AIS ≥ 4), accounting for 11.21%. The proportions of severe abdominal injuries in BAT and PAT patients were not significantly different (*P*=0.57). The ISS was also retrieved, and 55.73% (209) of cases involved minor-to-moderate injury (ISS ≤ 16). A total of 134 patients (35.73%) had severe injury (16 ≤ ISS ≤ 25), and 32 patients (8.54%) had very severe injury (ISS > 25). The proportion of BAT patients with severe injury was significantly higher than that of PAT patients (*P*=0.001). Regarding injury causes among severe-injury patients, traffic accident injury was still the most common, with a total of 80 patients (50%), followed by high-fall injury (34 patients, 20.48%).

### 3.4. Timeliness of Treatment

The median prehospital interval time was 1.34 hours (1.02–2.03 hours). There was no significant difference in the prehospital interval between the PAT and BAT groups (*P*=0.902, 1.34 hours (1.03–2.03 hours) vs. 1.54 hours (0.34–3.10 hours)). The median injury-regional hospital times in BAT and PAT patients were 10.47 hours (5.18–22.51 hours) and 7.00 hours (3.80–15.38 hours), respectively, which were statistically significant (*P*=0.001). The median preoperative time in surgical patients was 2.58 hours (1.37–5.35 hours), and there was no significant difference between the BAT group and the PAT group (*P*=0.902). Among those with hollow viscus injuries, the injury-regional hospital time and preoperative time in the PAT group were notably shorter than those in the BAT group (injury-regional hospital time: 7.07 hours (3.99–13.85 hours) vs. 10.23 hours (6.00–21.59 hours), *P*=0.002; preoperative time: 2.81 hours (1.85–3.63 hours) vs. 3.02 hours (2.01–5.58 hours), *P*=0.047).

Further subgroup analysis of the rescue time was also performed (Table 3). In the AIS <4 group, the PAT subgroup had an obviously shorter interval than the BAT subgroup (7.00 hours (3.53–15.19 hours) vs. 12.00 hours (6.52–24.88 hours), *P*=0.001), whereas in the AIS ≥4 group, there was no difference between the two groups. Regarding the preoperative time, there was no significant difference between the AIS ≥4 group and AIS <4 group (*P*=0.093), and it was equally prevalent in the PAT subgroup and BAT subgroup (AIS ≥4: *P*=0.767; AIS <4: *P*=0.776). In the hemodynamic stability subgroup analysis, the injury-regional hospital time was significantly shorter in the hemodynamic instable group than in the hemodynamic stable group (3.31 hours (2.31–3.98 hours) vs. 10.10 hours (6.07–23.63 hours), *P*=0.001), as was the preoperative time (1.92 hours (1.07–2.58 hours) vs. 3.07 hours (1.92–7.80 hours), *P*=0.001).

### 3.5. Surgery Information

A total of 359 (64.92%) patients underwent surgical treatment; the operative procedures are shown in Table 1. Laparoscopic surgery was performed in 65 cases (18.11%), with 54 patients undergoing 2D laparoscopic surgery and 11 patients undergoing 3D laparoscopic surgery. A total of 37 patients with BAT and 28 patients with PAT underwent laparoscopic surgery; the proportion of patients undergoing laparoscopic surgery in the PAT group was significantly higher than that in the BAT group (16.47% vs 9.66%, *P*=0.04). Among the surgeries, 28 patients (43.08%) underwent exploratory laparoscopy only, and the remaining 37 patients underwent therapeutic surgery, including 25 patients who were converted to laparotomy, the conversion rate was 38.46%.

Thirty patients (8.36% of the total surgical population) received a second operation. Sixteen secondary operations were performed due to surgical complications, of which abdominal infection was the most common (8 cases), followed by bleeding complications (4 cases). The remaining 14 cases were scheduled for secondary surgery, including 9 cases for fracture internal fixation, 2 cases for skin grafting, and 3 cases for hepatobiliary or urinary surgery.

### 3.6. Postoperative Treatment and Prognosis

Thirty-nine patients (7.05%) were admitted to the intensive care unit (ICU) for further treatment without undergoing surgery, and 231 patients were admitted to the ICU after surgery, accounting for 64.35% of all surgical patients. The median postoperative ICU treatment duration was 4.00 days (2.00–10.00 days). Among them, 125 patients (46.30%) were treated for less than 3 days in the ICU and 33 patients (12.22%) were treated for more than 21 days in the ICU. The median postoperative hospital stay in patients with abdominal trauma cases was 10 days (6.00–21.00 days); 26.47% (95 patients) stayed less than 7 days, and 52.92% stayed more than 10 days, as shown in Figure 3.

As shown in Table 1, a total of 59 patients (10.66%) experienced complications during treatment, with 46 cases in the BAT group and 13 cases in the PAT group (*P* = 0.164). Further analysis, as shown in Figure 4, revealed that the highest incidence of complications was infection (47.46%), including 12 cases of surgery-related infections such as deep surgical site infections, wound infections, or ostomy infections, and 18 cases of nonsurgery-related infections such as pneumonia. The second most common complication among surgery-related complications was bleeding, with a total of 11 cases, followed by fistula (5) and obstruction (7).

In-hospital death occurred in 40 cases (7.23%). The main cause of death was multiorgan failure (MOF), followed by bleeding and severe infection. The overall 90-day mortality was 11.93% (66 cases), with 55 of the deaths occurring within 30 days. Among them, there were 18 cases in the PAT group and 48 cases in the BAT group, with no significant difference in mortality rate between the two groups. In the survival analysis (shown in Table 4), age, injury factors, injury-regional hospital time, AIS value, ISS value, multiple injuries, ICU care, and reoperation were associated with overall survival (*P* < 0.10). Further multivariate analysis showed that longer injury-regional hospital time (HR: 1.01, 95% CI: 1.00–1.02, *P*=0.008), severe ISS (ISS>25 vs. ISS<16, HR: 2.78, 95% CI: 1.380–5.60, *P*=0.004), and ICU treatment (with vs. without ICU treatment, HR: 4.69, 95% CI: 2.54–8.65, *P*=0.001) were independent risk factors for worse prognosis. The Kaplan‒Meier analysis for 90-day survival by trauma severity and ICU care is presented in Figure 5.

## 4. Discussion

Abdominal trauma is the third most common type of trauma, involving approximately one-third of the total trauma population. The overall mortality rate varies greatly among studies and regions, ranging from 6% to 36% [14–16]. Young people are the main population affected by abdominal trauma, which is the main cause of death and disability in this age group [17] and causes serious financial burdens on society and families. Therefore, it is of great significance to investigate the disease and treatment characteristics of abdominal trauma.

The overall in-hospital mortality rate in this cohort was 7.23%, and the most common factor causing death was multiple organ failure. Traffic injury was the most common cause of abdominal trauma, followed by sharp-object injury and high-fall injury, and these three factors were also the most common causes of serious injury. BAT accounted for the majority of abdominal injuries (69.26%), which was consistent with reports in previous research [18, 19]. In terms of injured organs, the most common three types of injuries were spleen (22.67%), liver (20.30%), and small bowel (17.01%) injuries. Among BAT patients, spleen and liver accounted for the highest two proportions [16, 18, 20], whereas the most prevalent site of injury in PAT patients was the small intestine and colon, which differed from the findings in other studies. In a study of abdominal trauma in Mexico, the small intestine was the most commonly injured organ, followed by the liver and colon [16], and similar conclusions were reported in relevant studies in Europe, where small intestinal injury and liver injury were the most common injuries, accounting for up to approximately 30% of abdominal injuries [6, 21]. The reasons for the difference were mainly related to the different backgrounds of trauma. In this study, firearm injury accounted for only 1.45% (8 cases), which might also be the reason that the proportion of PAT patients with minor injury was significantly higher than that of BAT patients (*P*=0.001). Hollow viscus injury accounted for 41.22% of all patients in this study, and this proportion was relatively high compared with those in previous studies, ranging from 6% to 40% [15, 16, 18, 21]. In this study, hollow viscus injury accounted for 37.07% of BAT injuries, and there were mainly two reasons for the high proportion of hollow viscus injuries: First, the treatment of solid organ injury in hemodynamically stable patients relies mainly on nonsurgical treatment, and this concept has been increasingly recognized [22, 23]. Some patients with kidney (90%), spleen, and liver (70–80%) injuries can be treated and recovered with nonsurgical therapy [24]. This means that a large proportion of solid organ injuries can be treated in local hospitals without transfer to a regional medical center. Second, the diagnosis and management of hollow viscus injury in BAT is still a difficult problem, and currently available examination and diagnostic methods make it challenging to determine whether surgical intervention is necessary, and delayed surgery may lead to higher mortality. Such patients usually have multiple organ injuries, and their condition is relatively complex [6, 11, 23–25]. Therefore, although BAT patients with suspected hollow viscus injury are more likely to be transferred to regional medical centers, the rescue time between injury and arrival at a regional medical center was significantly higher in BAT patients than in PAT patients.

Compared with that in 2010–2015, the number of cases transferred from surrounding areas to regional medical centers was significantly smaller in the latter 6 years, which is presumed to be closely related to the gradual completion of the prehospital emergency transport system in China. One regional trauma medical center with several secondary hospitals and rescue stations in a region was established to reduce the time and resources required for the cross-regional transport of trauma patients [26]. In this study, the median prehospital time was 1.34 hours, while the median injury-regional hospital time was 9.7 hours because many patients were initially transported to the secondary medical center. More patients with BAT than those with PAT were transported to Beijing (*P*=0.008), which demonstrates the difficulty of diagnosis and treatment in BAT. The injury-regional hospital time was significantly shorter in the PAT group than in the BAT group (*P*=0.001). The reason for this difference is that PAT is easier to identify, and the decision to transfer can be made more quickly than that required for BAT. In BAT patients, asymptomatic hollow viscus injury is difficult to identify by physical or imaging examination, and the therapeutic strategy tends to be more conservative. In our results, the injury-regional hospital time and preoperative time in the hollow viscus injury BAT group were both significantly longer than those in the PAT group (*P*=0.002, *P*=0.047). By multivariate analysis, a longer injury-regional hospital time was shown to be an independent risk factor for worse prognosis. Therefore, more attention should be given to the treatment of BAT.

In the survival analysis, the prehospital transit time was not a significant risk factor for mortality (*P*=0.760). A recent literature meta-analysis reported that the length of prehospital stay was not significantly associated with mortality in younger or older trauma patients [27], which is consistent with our results. However, for hemodynamically unstable trauma patients, urgent systemic resuscitation and treatment are still crucial [28], and a rescue delay of more than 1.5 hours might increase the mortality risk by 70% [29]. At present, there are various treatment modalities for trauma among medical centers in China depending on their own situations and characteristics [30]. The use of a trauma management team or system to control and guide the timeliness of each trauma treatment procedure [31] can potentially shorten the prehospital and preoperative times in abdominal trauma treatment and improve patients' clinical outcomes.

Regarding treatment strategies, a total of 359 patients underwent surgical therapy. Small intestinal repair, stoma surgery and resection accounted for the largest proportions of all operations, and hollow viscus-related surgery was most common in patients with abdominal trauma. This suggests that trauma surgery training courses may need to include more general surgery-related skills, especially because the majority of abdominal trauma surgeries involve hollow viscus-related surgery [20]. In previous reports, hemorrhagic shock was the leading cause of death in patients with abdominal trauma [32]. In our cohort, bleeding was the second leading cause of death; this difference may be related to the low proportion of gunshot and sharp-object injuries in our study.

In the case of patients with PAT, a previous report showed that only 50–70% of abdominal stab injuries penetrate the peritoneum, and only 50–70% require surgical intervention [9]. For hemodynamically stable penetrating injuries, the latest WSES guidelines recommend the routine use of local wound exploration (LWE), laparoscopic exploration, or laparotomy for diagnosis [33], an approach also reflected in gunshot injury treatment guidelines [34]. Laparoscopic exploration procedures in trauma have been gradually standardized [35], and recent research has demonstrated a low false-negative rate of only 1.4% in laparoscopic exploration for abdominal trauma patients [36]. Our team previously conducted a small multicenter study to demonstrate the safety of laparoscopy in the treatment of abdominal trauma; we also found a significantly shorter average hospital stay compared with that for laparotomy [37]. In this study, laparoscopic exploration surgery was performed in 15 cases with suspicious abdominal wall penetrating injuries, effectively avoiding unnecessary laparotomy. As shown in Table 2, among hemodynamically stable patients, the proportion of hollow viscus injuries was significantly higher in the BAT group. However, the rate of laparoscopic surgery was significantly higher in the PAT group compared to the BAT group. The main reason is that the diagnosis and surgical decision-making for hollow viscus injuries in PAT are more challenging compared to penetrating trauma. For suspected hollow viscus and diaphragm injuries due to BAT, abdominal ultrasound and CT suffer from a high false-negative diagnosis rate of 20–40% [38, 39]. Accumulating evidence indicates that laparoscopic exploration might serve as an alternative method to confirm suspected hollow viscus injury when intra-abdominal injury cannot be totally ruled out [35]. Therefore, we believe that prompt laparoscopic exploration may be more beneficial for patients with persistent suspicion of hollow viscus injuries but without definitive evidence in BAT. However, further large-scale prospective studies are needed to validate this approach.

ICU treatment is an important part of abdominal trauma treatment. In this study, 64.35% of postoperative patients underwent ICU treatment, and ICU treatment was an independent risk factor for mortality (*P*=0.001). The median postoperative hospital stay was 10 days (6.00–21.00 days), and 52.92% of patients had a postoperative hospital stay of more than 10 days, which was even higher in patients with other comorbidities. Longer hospitalization not only increases the financial burden on patients but also increases the incidence of in-hospital complications [40]. Only 20% of prolonged hospital stays are related to medical treatment [41], and the major factor for the prolongation of hospitalization is a lack of appropriate rehabilitation institutions for trauma patients, followed by postoperative complications. In this study, a total of 59 patients experienced complications during hospitalization, with 16 cases (27.12%) requiring secondary surgery, accounting for 53.3% of all reoperation cases. Thus, it is necessary to focus on the quality of surgical procedures and address unsafe factors after stabilizing a patient's condition.

There are also several limitations of this study. First, selection bias due to inclusion and exclusion criteria cannot be ignored. Although the clinical characteristics and treatment data were mainly objective, further prospective studies are still needed to confirm our findings. Second, some detailed information, e.g., blood test results, injury posture in traffic or high-fall trauma, is lacking, which compromised our analytic results. Furthermore, longer prognostic data of trauma patients categorized by different trauma types or treatment are not available due to the lack of a follow-up registry in China.

## 5. Conclusion

Compared with PAT, the BAT group had a significantly higher proportion of patients with hollow viscus injuries in the hemodynamically stable subgroup. Additionally, more patients with BAT were transferred to higher-level hospital, resulting in significantly longer prehospital and preoperation time. In order to expedite patients receiving the correct treatment, aggressive diagnostic and investigative strategies may be beneficial, such as early laparoscopic exploration. Patients with prolonged injury-regional hospital times, severe ISSs, and a need for ICU care may have higher mortality.

## Figures and Tables

**Figure 1:** Selection flowchart.

**Figure 2:** The geographical distribution of enrolled patients.

**Figure 3:** ICU stays and postoperative hospital stays.

**Figure 4:** Complications encountered during treatment.

**Figure 5:** Kaplan–Meier survival plot for abdominal trauma patients. (a) 90-day survival in overall population; (b) 90-day survival by ISS scores; (c) 90-day survival by ICU treatment.

**Table 1:** Organ injuries treated by surgery and procedures.

Identified organ injuries and procedures		Penetrating abdominal trauma	Blunt abdominal trauma
Identified organ injuries	547	146	401
Solid organs (*n*%)	295 (53.93)	41 (28.08)	254 (63.34)
Liver (*n*%)	122 (22.30)	20 (13.70)	102 (25.44)
Interventional therapy	33	0	33
Hepatorrhaphy	36	10	26
Hepatectomy	24	10	14
Hemostassis and drainage	29	0	29
Spleen (*n*%)	124 (22.67)	11 (7.53)	113 (28.18)
Interventional therapy	21	0	21
Splenorrhaphy	16	3	13
Splenectomy	77	8	69
Hemostassis and drainage	10	0	10
Pancreas (*n*%)	44 (8.04)	7 (4.79)	37 (9.27)
Hemostassis and drainage	33	5	28
Distal pancreatectomy	11	2	9
Kidney (*n*%)	5 (0.91)	3 (2.05)	2 (0.49)
Nephrectomy	2	1	1
Nephrorrhaphy	3	2	1
Hollow organ (*n*%)	183 (33.46)	87 (59.60)	96 (23.94)
Stomach (*n*%)	30 (5.48)	24 (16.44)	6 (1.50)
Primary closure of stomach	30	24	6
Small bowel (*n*%)	93 (17.01)	34 (23.29)	59 (14.70)
Primary closure of small bowel	60	28	32
Bowel resection and anastomosis	33	6	27
Colorectum (*n*%)	60 (10.97)	29 (19.86)	31 (7.72)
Primary closure of colon	26	14	12
Repair or resection and ostomy	34	15	19
Mensenterium, omentum, peritoneum and diaphragm (*n*%)	55 (10.05)	13 (8.91)	42 (10.46)
Ligation of bleeder and repair	47	12	35
Bowel resection and anastomosis	8	1	7
Ureter and urinary bladder (*n*%)	14 (2.57)	5 (3.43)	9 (2.24)
Primary closure of ureter/urinary bladder	11	5	6
Cystostomy or nephrostomy	3	0	3

**Table 2:** Clinical characteristics of enrolled abdominal trauma patients.

	All patients	Penetrating abdominal trauma	Blunt abdominal trauma	PAT vs BAT
				*P* value
*Age (years, n%)*				
<18	38 (6.87)	13 (7.65)	25 (6.53)	0.002
18–44	339 (61.31)	122 (71.77)	217 (56.66)	
45–59	124 (22.42)	27 (15.88)	97 (25.33)	
>59	52 (9.40)	8 (4.70)	44 (11.49)	
*Sex*				
Male	481 (86.80)	151 (88.82)	330 (86.16)	0.391
Female	72 (13.20)	19 (11.18)	53 (13.84)	
*Injury factor (n%)*				
Traffic accident injury	225 (40.69)	5(2.94)	220 (57.44)	0.001
High fall injury	71 (12.84)	6 (3.53)	65 (16.97)	
Mechanical injury	25 (4.52)	10 (5.88)	15 (3.92)	
Sharps injury	137 (24.77)	137 (80.59)	0	
Fall injury	29 (5.24)	1 (0.59)	28 (7.31)	
Firearm injury	8 (1.45)	8 (4.71)	0	
Other violent injuries	58 (10.49)	3 (1.76)	55 (14.36)	
*AIS value (n%)*				
1	44 (7.96)	23 (13.52)	21 (5.48)	0.019
2	160 (28.93)	47 (27.65)	113 (29.50)	
3	287 (51.90)	79 (46.47)	208 (54.31)	
4	54 (9.76)	19 (11.18)	35 (9.14)	
5	8 (1.45)	2 (1.18)	6 (1.57)	
*Severe abdominal trauma (AIS ≥ 4, n%)*				
AIS < 4	491 (88.79)	149 (87.65)	342 (89.30)	0.570
AIS ≥ 4	62 (11.21)	21 (12.35)	41 (10.70)	
*ISS value (n%)*				
<16	209 (55.70)	112 (72.26)	97 (44.09)	0.001
16–25	134 (35.70)	38 (24.52)	96 (43.64)	
>25	32 (8.60)	5 (3.23)	27 (12.27)	
Initial systolic blood pressure (mmHg)	119 (100–136)	118.5 (101–113.30	120 (99–137)	0.853
Initial heart rates	104.70 ± 20.23	105.4 ± 19.99	103.00 ± 20.73	0.187
Initial hemoglobin (mg/dl)	121 (101–142.50)	130 (111.50–147.00)	118 (99.00–139.00)	0.001
Lactate (mmol/L)	2.40 (1.50–3.45)	2.50 (1.38–3.70)	2.30 (1.60–3.40)	0.780
Potential of hydrogen (PH)	7.32 ± 0.13	7.32 (7.22–7.40)	7.31 ± 0.13	0.680
Hemodynamic stability (*n*%)	476	134	342	
Solid organ injury	282	61	221	0.001
Hollow viscus injury	158	60	98	
Solid & hollow organ injury	36	13	23	
Hemodynamic instability (*n*%)	62	21	41	
Solid organ injury	28	8	20	0.718
Hollow viscus injury	28	11	17	
Solid & hollow organ injury	6	2	4	
Laparoscopy surgery (*n*%)	65 (18.11)	28 (16.47)	37 (9.66)	0.044
Mortality (*n*%)	66 (11.93)	18 (10.59)	48 (12.53)	0.335
Complications (*n*%)	59 (10.66)	13 (7.65)	46 (12.01)	0.164

**Table 3:** Timeliness of abdominal trauma treatment.

Groups	Injury-reginal hospital time median (IQR) (h)	*P* value	Preoperative time median (IQR) (h)	*P* value
Blunt abdominal trauma	10.47 (5.18–22.51)	0.001	2.55 (1.27–6.42)	0.902
Penetrating abdominal trauma	7.00 (3.80–15.38)		2.80 (1.88–4.25)	
Hollow viscus injury (in BAT)	10.23 (6.00–21.59)	0.002	3.02 (2.01–5.58)	0.047
Hollow viscus injury (in PAT)	7.07 (3.99–13.85)		2.81 (1.85–3.63)	
AIS ≥ 4	9.55 (6.00–18.51)	0.862	2.82 (1.35–6.50)	0.093
AIS < 4	10.00 (5.00–21.60)		2.67 (1.46–5.22)	
BAT (AIS ≥ 4)	7.8 (4.00–17.29)	0.604	2.48 (1.37–6.66)	0.767
PAT (AIS < 4)	10.36 (5.00–17.18)		3.00 (2.00–7.00)	
BAT (AIS < 4)	12.00 (6.52–24.88)	0.001	2.55 (1.23–6.92)	0.776
PAT (AIS < 4)	7.00 (3.53–15.19)		2.79 (1.86–4.03)	
ISS < 16	10.00 (5.00–20.95)	0.840	2.80 (1.65–5.20)	0.335
25 > ISS ≥ 16	10.00 (5.08–23.11)		2.50 (1.32–5.58)	
ISS ≥ 25	10.08 (6.74–18.83)		2.00 (1.08–7.16)	
Hemodynamic stability	10.10 (6.07–23.63)	0.001	3.07 (1.92–7.80)	0.001
Hemodynamic instability	3.31 (2.31–3.98)		1.92 (1.07–2.58)	

**Table 4:** Univariate and multivariate analyses for 90 days survival after abdominal trauma.

Factor	Univariate analysis		*P* value	Multivariate analysis		*P* value
	HR	95% CI		HR	95% CI	
Sex			0.813			
Male	1.00					
Female	1.09	0.54–2.20				
Age (y)						
<18	1.00			1.00		
18–44	1.65	0.40–6.91	0.491	0.94	0.22–4.02	0.932
45–59	2.82	0.66-12.05	0.163	1.58	0.36–6.90	0.542
>59	4.86	1.10–21.52	0.037	2.66	0.59-12.12	0.205
Injury factor						
Traffic accident injury	1.00					
High-fall injury	0.69	0.31–1.57	0.378			
Mechanical injury	0.87	0.27–2.86	0.823			
Sharp-objects injury	0.59	0.30–1.17	0.132			
Fall injury	0.74	0.23–2.42	0.619			
Firearm injury	3.19	0.98-10.43	0.054			
Other violent injuries	0.78	0.35–1.77	0.557			
Prehospital transit-time	0.93	0.59–1.47	0.760			
Injury-reginal hospital time	1.01	1.01–1.02	0.025	1.01	1.00–1.02	0.008
Preoperative time	0.99	0.95–1.03	0.518			
AIS value						
<4	1.00					
≥4	2.37	1.31–4.28	0.004			
ISS value						
<16	1.00			1.00		
16–25	1.21	0.68–2.18	0.515	0.79	0.43–1.44	0.437
>25	4.55	2.38–8.72	0.001	2.78	1.38–5.60	0.004
Trauma category						
PAT	1.00					
BAT	0.85	0.49–1.45	0.545			
Multiple injuries						
Yes	3.25	1.61–6.57	0.001			
No	1.00					
Surgery treatment						
Yes	1.23	0.92–1.65	0.170			
No	1.00					
ICU treatment						
Yes	2.23	1.67–2.98	0.001	4.69	2.54–8.65	0.001
No	1.00			1.00		
Reoperation						
Yes	2.79	1.12–6.91	0.027			
No	1.00					

## Data Availability

All data from which the conclusion could be drawn are presented in the manuscript. No additional data are available.
